# Construction and Validation of a Prognostic Model Based on mRNAsi-Related Genes in Breast Cancer

**DOI:** 10.1155/2022/6532591

**Published:** 2022-10-11

**Authors:** Xugui Zhao, Jianqing Lin

**Affiliations:** Department of Thyroid and Breast Surgery, The Second Affiliated Hospital of Fujian Medical University, Quanzhou 362000, China

## Abstract

**Background:**

Breast cancer is a big threat to the women across the world with substantial morbidity and mortality. The pressing matter of our study is to establish a prognostic gene model for breast cancer based on mRNAsi for predicting patient's prognostic survival.

**Methods:**

From The Cancer Genome Atlas (TCGA) and Gene Expression Omnibus (GEO) databases, we downloaded the expression profiles of genes in breast cancer. On the basis of one-class logistic regression (OCLR) machine learning algorithm, mRNAsi of samples was calculated. Kaplan-Meier (K-M) and Kruskal-Wallis (K-W) tests were utilized for the assessment of the connection between mRNAsi and clinicopathological variables of the samples. As for the analysis on the correlation between mRNAsi and immune infiltration, ESTIMATE combined with Spearman test was employed. The weighted gene coexpression network analysis (WGCNA) network was established by utilizing the differentially expressed genes in breast cancer, and the target module with the most significant correlation with mRNAsi was screened. Gene Ontology (GO) and Kyoto Encyclopedia of Genes and Genomes (KEGG) analyses were conducted to figure out the biological functions of the target module. As for the construction of the prognostic model, univariate, least absolute shrinkage and selection operator (LASSO) and multivariate Cox regression analyses were performed on genes in the module. The single sample gene set enrichment analysis (ssGSEA) and tumor mutational burden were employed for the analysis on immune infiltration and gene mutations in the high- and low-risk groups. As for the analysis on whether this model had the prognostic value, the nomogram and calibration curves of risk scores and clinical characteristics were drawn.

**Results:**

Nine mRNAsi-related genes (CFB, MAL2, PSME2, MRPL13, HMGB3, DCTPP1, SHCBP1, SLC35A2, and EVA1B) comprised the prognostic model. According to the results of ssGSEA and gene mutation analysis, differences were shown in immune cell infiltration and gene mutation frequency between the high- and low-risk groups.

**Conclusion:**

Nine mRNAsi-related genes screened in our research can be considered as the biomarkers to predict breast cancer patients' prognoses, and this model has a potential relationship with individual somatic gene mutations and immune regulation. This study can offer new insight into the development of diagnostic and clinical treatment strategies for breast cancer.

## 1. Introduction

Breast cancer is a common threat to the women with increased annual incidences, and it has surpassed lung cancer ranking 1st on the global cancer-statistics list in 2020 [1]. Usually, the factors to assess the conditions of breast cancer patients lie in tumor stage, histological grade, and molecular subtype. However, when it comes to the prediction of patients' prognoses, they just do little help regarding the accuracy [2]. Prediction based solely on pathological features is likely to cause inaccurate diagnosis of patient's prognosis. For one thing, low low-risk patients are likely to undergo unnecessary or excessive treatment. For another, the improper treatment tends to put high-risk patients as risk of cancer recurrence or metastasis [3]. For example, He et al. [4] explored SNP-related genes as novel prognostic markers for breast cancer, whose predictive performance for either disease-free survival or prognostic risk of patients is difficult to be realized by other clinicopathological characteristics. As a result, to explore novel biomarkers capable of predicting breast cancer patient's prognosis is of great significance for treating patients with more precise therapeutic strategies.

The complexity and diversity in tumor microenvironment are beyond our imagination. Some cells are responsible for tumor initiation, metastasis, and recurrence in tumor microenvironment, but others are not. For a few cells with stemness features and invasiveness, they can trigger the development of tumor and invade human immune system, inducing innate resistance to external killing [5, 6]. These cells are named as cancer stem cells (CSCs), which have the features of continuous proliferation, self-renewal, and multidirectional differentiation [4]. Breast cancer stem cells can induce various primary tumors, facilitating the development and metastasis of tumors, resulting in a poor prognostic response in breast cancer patients [7]. Notably, multiple CSC-associated breast cancer molecular markers have been identified, such as CD44, CD24, ALDH1, PROCR, and MUC1 [8, 9]. Among them, CD44, CD24, and ALDH1 are capable of predicting the prognoses of triple-negative breast cancer patients, which can be predictive markers for cancer recurrence, distant metastasis, disease-free survival, and overall survival [10, 11]. Revealing breast cancer prognostic markers from the perspective of CSCs may be an important entry point.

Given the important regulation of CSC properties for tumor progression, existing studies have established a new method to describe CSCs through machine learning algorithms capable of quantifying the differentiation phenotype during cancer progression and the development characteristics of stem cell populations in tumor tissues [12]. For the identification of various stem cells and tumor cells, the one-class logistic regression (OCLR) machine learning algorithm is a great choice utilized to extract the expression profiles of these cells [13]. The algorithm has been applied to the genome-wide expression data of enormous TCGA samples and successfully quantified the differentiation degree of various cancers of the breast cancer, lung cancer, glioma, and so on, as well as the stemness features and tumorigenicity of paired healthy tissues. Finally, a new stemness feature mRNAsi was proposed [13]. mRNAsi is a cancer stem cell index describing the similarity degree between tumor and stem cells, which can be considered a quantification of cancer stem cells [13]. The values of mRNAsi range from 0 to 1, and it has a close connection with the tumor dedifferentiation level and biological processes of CSCs [14, 15]. mRNAsi has been verified as an indicator of survival, classification, and disease progression in cancer patients [15–17]. Above-mentioned studies have paved the way for us to dive deeper into the mechanisms of breast cancer stem cells and the mining of prognostic molecular markers. The epigenetically regulated mRNA expression-based stemness index (EREG-mRNAsi) is obtained by training the expression level of genes associated with the epigenetically regulated stem cells. The index ranges from 0 to 1. The closer the index value is to 1, the lower the degree of cell differentiation and the stronger the stemness features, reflecting the degree of dedifferentiation of cancer cells [18, 19].

Our study initially determined the mRNAsi of TCGA-BRCA dataset samples, predicted tumor purity, and abundance of stromal cells and immune cells within the tumor and analyzed the correlation of mRNAsi with immune infiltration. The target gene module associated with mRNAsi was screened by weighted gene coexpression network (WGCNA). Next, a bioinformatics analysis on the target module revealed 9 mRNAsi-related genes that were capable of predicting breast cancer patient's prognosis, and a prognosis-assessing model was hence established. Subsequently, the study revealed the complex role of prognostic signature genes with somatic gene mutations and immune cell infiltration, providing a reference for the expansion of the prediction field of prognostic models. To sum up, the risk assessment model constructed in our study was able to effectively predict the prognosis of patients with breast cancer. Besides, the connection between 9 mRNAsi-related genes and somatic gene mutations as well as immune regulation was revealed in our study. These mRNAsi-related genes can be applied as biomarkers with great value in clinical practice like predicting prognoses of breast cancer patients.

## 2. Materials and Methods

### 2.1. Breast Cancer Sample Data Collection

From TCGA database (https://portal.gdc.cancer.gov/), breast cancer RNA expression data, gene mutation data, and corresponding clinical data were obtained as training sets, involving 1109 breast cancer samples and 113 healthy breast samples. From the EGB (http://asia.ensembl.org/index.html), the GTF annotation file was acquired. From the GEO library (https://www.ncbi.nlm.nih.gov/geo/), the breast cancer sample expression profile GSE42568 (https://www.ncbi.nlm.nih.gov/geo/query/acc.cgi? acc = GSE42568) was downloaded as the validation set. The mRNAsi of samples was calculated by OCLR [13] for the comparison of the mRNAsi differences between the normal and tumor groups.

### 2.2. Correlation between Stemness Index of mRNAsi and Clinicopathological Variables and Immune Infiltration

Overall survival was compared between different mRNAsi samples by Kaplan-Meier (K-M) analysis according to the optimal threshold. The R package ggpubr (https://cran.r-project.org/web/packages/ggpubr/index.html) was employed for comparing mRNAsi in the context of clinical characteristics. The Kruskal-Wallis (K-W) test was employed for assessing the connection between mRNAsi and clinical characteristics. Based on the gene expression profiles of breast cancer samples, ESTIMATE was utilized to generate immune, stromal, and ESTIMATE scores, as well as tumor purity. The correlation analysis on mRNAsi and these scores and tumor purity were achieved by Spearman's test, and *p* values were calculated.

### 2.3. WGCNA

FPKM data from TCGA-BRCA were identified for differentially expressed genes (DEGs) utilizing the R package limma [20] (|log2FC| > 1, FDR < 0.05). On the basis of these DEGs, the R package WGCNA was utilized for the analysis of the Gene modules [21], and the specific processes were as follows: genes with missing values were removed using the goodSamplesGenes function, tumor samples were clustered, outliers were removed, and 100 was set as a cut line. The coexpression network was constructed by setting 6 as the optimal soft threshold. Then, by transforming the adjacency matrix into a TOM matrix, the genetic connectivity of the network was detected. Next, the average linkage hierarchical clustering was performed on the basis of the differences in TOM. By employing a dynamic shearing approach, the gene tree was then divided into different modules. And the minimum number of genes in each module was set to 50, and MEDissThres was set at 0.25 to cluster and merge similar modules.

### 2.4. Gene Function Annotation of Gene Module

In each gene module, there was a primary component, namely, module eigengenes (MEs) which could represent all genes within the module. To mine the gene modules associated with mRNAsi of tumor samples, the ME of each module was calculated separately with the mRNAsi of the samples for correlation coefficient, and the gene modules highly associated with mRNAsi were retained as the target modules. The R package clusterProfiler [22], enrichplot (https://bioconductor.org/packages/release/bioc/html/enrichplot.html), and ggplot2 (https://ggplot2-book.org/) were utilized for the annotation and visualization of KEGG and GO pathways.

### 2.5. Construction and Validation of the Prognostic Model

The R package survival (https://cran.r-project.org/web/packages/survival/index.html) was used to perform univariate Cox regression analysis on genes in the target module to identify genes that have a close connection with patient's overall survival rate (*p* < 0.01). The R package glmnet [23] and survival were utilized for the conduction of LASSO analysis, which was combined with multivariate Cox analysis to further screen genes and risk coefficients remarkably linked to prognosis, thus to construct a risk model. Data from TCGA-BRCA was classified as high- and low-risk groups taking the median risk score as a demarcation. Differences in mRNAsi between the two groups were analyzed employing the R package ggpubr, and K-M curves and ROC curves were plotted employing the R package survival. At last, the risk score, survival state plots, and gene expression heat map of the two risk groups was plotted.

### 2.6. Analysis of the Correlation between Prognostic Models and Tumor Immunity and Gene Mutations

The R package GSEABase with 29 immune-related features [24] was employed for the conduction of ssGSEA analysis of genes in the prognostic risk assessment model. By utilizing the R package heat map, the antitumor immune-enrichment results of the high- and low-risk groups were visualized. In gene mutation analysis, R package maftools [25] was utilized for analyzing the tumor mutational burden, and R package GenVisR [26] was utilized for analyzing the differences in gene mutation types and mutation numbers of the samples.

### 2.7. Prognostic Model Validity Assessment

In this study, univariate and multivariate Cox regression analyses of risk score, age, gender, pathological stage, and other clinical characteristic parameters were conducted utilizing the R package survival in TCGA-BRCA or GSE42568 datasets. The R packages rms, regplot, tibble, and survival were used to draw nomograms according to the risk score and 6 clinicopathological factors. Calibration curve was drawn to predict the consistency between nomogram-predicted 1-, 3-, and 5-year survival and actual survival of patients.

## 3. Results

### 3.1. Breast Cancer mRNAsi Is Closely Bound Up with the Clinical Characteristics of Patients and Immune Regulation of Cancer Tissues

mRNAsi can reflect the similarity between tumor cells and stem cells. In this study, differential analysis of breast cancer samples with mRNAsi data and corresponding healthy breast samples demonstrated that mRNAsi was substantially upregulated in breast cancer tissues (Figure 1(a)). Samples were classified into high- and low-risk groups according to the optimal threshold of mRNAsi. Survival analysis illustrated that a higher mRNAsi index in patients led to a poorer prognostic survival rate with a contrast to that of patients with a lower mRNAsi index (Figure 1(b)). Patients with higher EREG-mRNAsi had poorer overall survival compared with patients with lower EREG-mRNAsi (Figure 1(c)). Correlation analysis between mRNAsi and clinicopathological characteristic variables of breast cancer showed that mRNAsi expression did not significantly change with tumor growth (Figure 1(d)) but was significantly increased with the progression of pathological stage (Figure 1(e)). Given the potential role of mRNAsi in the antitumor immune process, this study speculated that mRNAsi added much diversity to the tumor immune microenvironment. Therefore, the construction of correlation between the ESTIMATE assessment results of TCGA-BRCA tissues with the mRNAsi of the samples told us that mRNAsi was negatively correlated with the stromal score, immune score, and ESTIMATE score of tumor tissues. But a positive correlation was found in mRNAsi with tumor purity (Figures 1(f)–1(i)). The finding revealed a close connection between breast cancer mRNAsi and the clinical characteristics of patients and the immune regulation of cancer tissues. This index was worthy of inclusion in subsequent studies to reveal its biological function.

### 3.2. Identification of mRNAsi-Related Modules

In view of the significant difference in mRNAsi between normal and tumor tissues, we first screened DEGs from the mRNA level to elucidate differences in mRNAsi, which were visualized in a volcano plot (Figure 2(a)). To dig out key mRNAsi-related genes, WGCNA was conducted for the construction of a coexpression network of mRNAs for TCGA-BRCA. The index of the scale-free topology was taken to reach 0.90 (Figures 2(b) and 2(c)). By using a dynamic tree pruning algorithm (module size = 50), genes with similar expression patterns were introduced into the same module to form a hierarchical clustering tree with modules. According to the weighted correlation and the set criteria, hierarchical clustering analysis was performed, and clustering results were segmented (Figure 2(d)). Six gene modules were finally identified, and correlation analysis of MEs with mRNAsi and EREG-mRNAsi in each module revealed that the blue module presented the highest correlation with cell stemness index mRNAsi (*r* = 0.74, *p* = 1*e* − 190) (Figure 2(e)). As shown in Figure 2(f), among the blue module genes, the closer module membership value is to 1 indicates that the gene is more strongly correlated with this module. The higher value of gene significance for mRNAsi indicates that mRNAsi is more correlated with the gene in the module. As a result, we adopted the blue module with 385 genes as the target module for subsequent studies.

### 3.3. Gene Function Annotation of Target Module

To investigate how mRNAsi-related genes and pathways functioned biologically, GO functional annotation and KEGG pathway enrichment analyses were performed on 385 genes from the target blue module. GO functional annotation results indicated that these genes were primarily bound up with functions including chromosome segregation, organelle fission, and nuclear division (Figure 3(a)). KEGG pathway enrichment analysis suggested that the involvement of these genes was found in cell cycle, human T cell leukemia virus 1 infection, and oocyte meiosis (Figure 3(b)). GO and KEGG results showed that genes of the blue module were mainly enriched in signaling pathways associated with cell cycle, T cell leukemia virus, and oocyte division, which are closely related to cancer development.

### 3.4. Establishment of the mRNAsi-Based Prognostic Model

Firstly, the prognostic effect of the genes in the blue module was assessed by the univariate Cox regression analysis. Then, 9 candidate feature genes were screened by the LASSO Cox regression analysis under the optimal value of *λ* (Figures 4(a) and 4(b)). The risk assessment model was finally constructed based on 9 genes, through multivariate Cox regression analysis (Figure 4(c)). Risk score = −0.0725^∗^CFB + 0.1894^∗^MAL2 − 0.4245^∗^PSME2 + 0.0826^∗^MRPL13 + 0.0736^∗^HMGB3 + 0.3917^∗^DCTPP1 + 0.0628^∗^SHCBP1 + 0.1012^∗^SLC35A2 − 0.0566^∗^EVA1B.

TCGA-BRCA samples were divided into high- and low-risk groups by setting the median risk score as the cutoff value, and the heat map showed the expression levels of 9 mRNAsi-related genes (Figure 4(d)). The distribution of risk score and survival time among samples in TCGA dataset showed that as risk score increased, the mortalities from cancer also mounted and the survival time decreased (Figures 4(e) and 4(f)). Differential analysis of mRNAsi demonstrated that patients in the high-risk group had markedly higher mRNAsi than those in the low-risk group (*p* = 6.732*e* − 27) (Figure 4(g)). Survival analysis demonstrated that high-risk group patients had a remarkably lower overall survival rate than low-risk group patients (*p* < 0.001) (Figure 4(h)). ROC curves demonstrated that the AUC values of the risk assessment model for predicting 1-year, 3-year, and 5-year survival of TCGA dataset samples were 0.71, 0.68, and 0.70, respectively (Figure 4(i)). The AUC values of the model for predicting 1-year, 3-year, and 5-year survival of GSE42568 dataset samples were 0.9, 0.67, and 0.74, respectively (Figure 4(j)). It was shown that the risk score for constructing a risk assessment model based on the 9 mRNAsi-related genes obtained from TCGA-BRCA dataset had predictive potential for breast cancer patients.

### 3.5. Immunological Infiltration and Gene Mutation Revelation in High- and Low-Risk Groups

We inferred the immune cell infiltration level in the breast cancer gene set by ssGSEA, and the expression level of immune gene set in the low-risk group was higher compared with the high-risk group (Figure 5(a)). Simultaneous tumor mutation burden (TMB) analysis showed that TMB values demonstrated higher in high-risk patients (*p* = 9.3*e* − 06) (Figure 5(b)). Subsequently, further mutation gene analysis demonstrated that the high-risk group samples had a much higher gene mutation frequency than the low-risk group samples (Figures 5(c) and 5(d)). There are differences in genetic variants between high- and low-risk groups, contributing to the difference in patient prognosis or immune cell infiltration.

### 3.6. Construction and Evaluation of the Nomogram

Univariate Cox analysis of risk score and other pathological features in TCGA dataset showed that age, pathological stage, distant tumor metastasis (M), lymph nodes metastasis (N), and risk score were all bound up closely with the prognosis of breast cancer patients, with a HR of 1.714 (*p* < 0.001) for risk score (Figure 6(a)). Multivariate analysis demonstrated that the HR of risk score was 1.592 (*p* < 0.001) (Figure 6(b)), indicating that risk score could be used as a prognostic factor independent of clinical characteristics. The nomogram plotted in combination with risk score, T, N, M stage, sex, age, and stage was used to predict the overall survival rate at 1, 3, and 5 years in patients with breast cancer (Figure 6(c)), corresponding to a better fit of the calibration curve (Figure 6(d)), demonstrating that this nomogram had a favorable predictive ability.

## 4. Discussion

CSCs have gained much attention in the cancer-related research. The intensive findings about CSCs have enriched our understandings of cancer development, thus propelling us to explore novel effective therapeutic strategies for combating cancer [10, 27]. mRNAsi can reflect stemness in cancer patients. With the help of computational biology and bioinformatics, mRNAsi can be used efficiently for mining genes related to tumor stemness [12, 13]. Since then, there have been a number of studies applying mRNAsi to cancer prognosis. For example, it has been shown that mRNAsi expression in hepatocellular carcinoma increases with tumor pathological grade, and mRNAsi established from gene expression data has a deep connection with poor overall survival of hepatocellular carcinoma patients [28]. In glioblastoma, the mRNAsi index of cancer tissue can be used to distinguish glioblastoma subtypes, and there is a marked difference in the prognostic overall survival rate of patients with each subtype [29]. The above reports all provide an important reference for the construction of predictive prognostic model for breast cancer based on mRNAsi.

Our study first established a correlation between TCGA-BRCA tissue assessment results and sample mRNAsi, and differentially expressed mRNAs were then obtained. Based on WGCNA mining the target modules closely related to mRNAsi, GO functional annotation and KEGG analyses of the genes in this module showed that they were mainly associated with functions such as chromosome segregation, organelle fission, and mitosis and were involved in cell cycle, human T cell leukemia virus 1 infection, and oocyte division pathways. It has been found in breast cancer, colon cancer, and ovarian cancer that the cell cycle mainly regulates specific transcription dependent on cell cycle genes in cancer [30–32]. Human T cell leukemia virus (HTLV-1) is a retrovirus isolated from human T cell tumors and induces cancer development through multiple mechanisms [33]. Oocyte division is also strongly associated with ovarian carcinogenesis [34]. Therefore, the above pathways are closely related to cancer. Nine feature genes were then selected by Cox regression analysis, and a prognostic model for breast cancer consisting of nine mRNAsi-related genes was constructed. The model involved CFB, MAL2, PSME2, MRPL13, HMGB3, DCTPP1, SHCBP1, SLC35A2, and EVA1B, of which CFB, PSME2, and EVA1B were used as cancer prognostic protective factors, and the remaining genes were used as prognostic risk factors. CFB is stably upregulated in various cancer tissues, and in studies of adenocarcinoma, this gene has been shown to alleviate cancer progression by activating cellular immune responses, consistent with the trend of this study in predicting progression of breast cancer [35]. PSME2 has been less studied in cancer, and reports indicate that this gene is a typical poor prognostic marker in renal cell carcinoma and promotes malignant tumor progression by inhibiting autophagy [36]. High expression of EVA1B is bound up closely with high infiltration levels of T cells, macrophages, and neutrophils in cancer tissues, and high expression of this gene implies poor prognosis in glioma patients [37]. This contrasts with our finding, perhaps PSME2 and EVA1B possess cancer specific, and whether the regulation of these two genes also involves autophagy and tumor immune regulation in this study remains to be further explored. The remaining genes exist as risk factors for cancer prognosis, and most of the genes have confirmed this in existing studies. For example, MAL2 and MRPL13 can inhibit tumor antigen presentation to drive breast cancer immune escape, and upregulation of two genes in breast cancer has been demonstrated to drive malignant progression of cancer [38, 39]. Similarly, HMGB3 is also a prototypical marker of breast cancer progression but worsens cancer progression primarily by promoting formation of breast layers of breast cancer cells [40, 41]. DCTPP1 is an oncogene regulated by the oncogenic factor miR-378a-3p, and this gene facilitates breast cancer cell proliferation through the interference of DNA repair signaling pathway [42, 43]. The phenomenon of overexpression of SHCBP1 in breast cancer has been studied, and cellular experiments have demonstrated that this gene directly regulates breast cancer cell proliferation and promotes the cell cycle [44]. SLC35A2 is associated with hypoxia-inducible factors, heat shock proteins, transcription factors, and DNA damage-associated signaling and is involved in the regulation of neutrophil and macrophage polarization in breast cancer [45]. In summary, the majority of the genes associated with mRNAsi of breast cancer in this study are closely related to cancer development or immune regulation of breast cancer, and it is reasonable to use this constructed prognostic model for clinical prognostic guidance.

In addition to uncovering the corresponding key genes, the results of ssGSEA analysis based on 9 mRNAsi genes in this study demonstrated that the difference regarding survival rate from the high-risk and low-risk group may originated from differences in immunoinfiltrating cells (e.g., Th2, CD8+ T cells, and NK cells). Th2 cells can secrete interleukins to participate in the body's humoral response and assist in the activation of human B cells and participate in antitumor immune responses. Downregulated infiltration of this cell in high-risk group predicts an immunosuppressive response, consistent with the results of this study. Similarly, this study revealed that CD8+ T cells downregulated in the TME act as the cells of choice for targeting cancer, activating cytotoxic T lymphocytes in the tumor immune circulation and mediating antitumor immune responses [46]. In clinical studies, NK cells often synergize with CD8+ T cells in antitumor immune processes, and both have similar cytotoxic mechanisms [47, 48]. This study revealed that the downregulation of multiple immune cell infiltration levels in the high-risk group was an indicator of an immunosuppressive microenvironment in this group, which might be the reason of the unsatisfactory prognosis discovered in high-risk group patients.

In summary, this study revealed the association between mRNAsi and clinical variables in breast cancer samples by K-M curve plotting and K-W test analysis. The gene modules associated with mRNAsi in breast cancer samples were constructed by WGCNA, which was used as a basis to screen and construct a 9-gene risk assessment model. The assessing performance this model on breast cancer patient's prognosis was also validated by WGCNA. ssGSEA analysis revealed the potential association of this risk model with individual somatic mutations and immune cell infiltration, which opens up new possibility for the development of diagnostic and clinical therapeutic strategies for treating breast cancer. However, this study is a bioinformatics analysis for model construction which is lack of clinical trials. Therefore, in future studies, we will collect more clinical sample data and incorporate some clinical information to increase the reliability of the model when constructing the model. At the same time, we did not use wet experiments to verify the constructed model, so we will perform relevant cellular experiments and molecular experiments to verify the model in subsequent experiments.

## Figures and Tables

**Figure 1:** Association between mRNAsi of TCGA-BRCA and clinical features and tumor immune microenvironment. (a) Differences in mRNAsi between TCGA-BRCA tissues and healthy samples. (b) K-M survival curve for mRNAsi. (c) K-M survival curve of EREG-mRNAsi. Tumor growth sizes in TCGA-BRCA tissue samples (d) and difference of mRNAsi expression in different clinical stages (e). (f–i) Correlation analysis between mRNAsi and stromal score (f), immune score (g), ESTIMATE score (h), and tumor purity (i) assessed by ESTIMATE algorithm.

**Figure 2:** Construction of weighted gene coexpression network of TCGA-BRCA samples. (a) Volcano plot showed the distribution of DEGs in breast cancer tumor tissue relative to normal breast tissue; red indicated upregulated genes, green indicated downregulated genes, and black indicated genes excluded by DEG screening criteria. (b) Scale-free topological model fit index screening. (c) Average connectivity of soft threshold of adjacency matrix. (d) Identification of breast cancer coexpressed gene modules; different colors represent different gene modules. (e) Heat map of correlation between gene modules and mRNAsi score or EREG-mRNAsi. (f) Scatter plot of blue gene modules; each circle represents a gene.

**Figure 3:** Blue module gene function annotation. (a) GO analysis of genes in the blue module. (b) KEGG pathway enrichment analysis of genes in the blue module; the color of the bubble represents the *p* value, and the size of the bubble represents the number of genes involved in the pathway.

**Figure 4:** Establishment of the mRNAsi-based prognostic model. (a) LASSO coefficient distribution of 14 prognosis-related genes. (b) Partial likelihood deviation calculated from LASSO regression cross-validation plotted as a function of log (*λ*). (c) Multivariate Cox analysis of 9 mRNAsi-related genes. (d) Heat map of gene expression for patients in high- and low-risk groups. (e) Risk score plot for patients in high- and low-risk groups. (f) Survival state diagram of patients in high- and low-risk groups. (g) Differential analysis of mRNAsi in patients in high- and low-risk groups. (h) K-M survival curves for patients in the high- and low-risk groups. (i) ROC curve of TCGA-BRCA sample to assess the predictive performance of the risk signature for 1-, 3-, and 5-year overall survival in the training set. (j) ROC curve of the GEO database GSE42568 dataset sample, used to assess the predictive performance of the 1-, 3-, and 5-year overall survival risk signature in the validation set.

**Figure 5:** Immune infiltration and gene mutation revelation in samples with different risk scores. (a) ssGSEA was used to infer the level of immune-infiltrating cells in the gene set of breast cancer samples from the high-risk and low-risk groups. (b) TMB differences between patients from the high-risk and low-risk groups. (c) Distribution of significantly mutated genes in breast cancer samples with mutations in the high-risk group. (d) Distribution of significantly mutated genes in breast cancer samples with mutations in the low-risk group, with different colors on the right side as different mutation types.

**Figure 6:** Construction and evaluation of nomogram. (a) Univariate Cox regression analysis of risk score and clinicopathological characteristics. (b) Multivariate Cox regression analysis of risk score and clinicopathological characteristics. (c) Nomogram constructed from risk score and clinicopathological characteristics to predict 1-, 3-, and 5-year survival rates of patients in the training cohort. (d) Calibration curve depicted the agreement between nomogram predicted 1-, 3-, and 5-year survival rates of patients and actual survival rates.

## Data Availability

The data used to support the findings of this study are available from the corresponding author upon request.
